RETRACTED

# The Reaction Pathway of miR-30c-5p Activates Lipopolysaccharide Promoting the Course of Traumatic and Hemorrhagic Shock Acute Lung Injury

**DOI:** 10.1155/2022/3330552

**Published:** 2022-04-13

**Authors:** Jianmin Li, Chanyuan Pan, Chao Tang, Wenwen Tan, Hui Liu, Jing Guan

**Affiliations:** ^1^Department of Pulmonary and Critical Care Medicine, Hunan Provincial People's Hospital, The First Affiliated Hospital of Hunan Normal University, Changsha, 410005 Hunan, China; ^2^Department of Science and Education, The First Hospital of Changsha, Changsha, 410008 Hunan, China

## Abstract

Acute lung injury (ALI) is an acute hypoxic respiratory failure caused by diffuse inflammatory injury in alveolar epithelial cells during severe infection, trauma, and shock. Among them, trauma/hemorrhagic shock (T/HS) is the main type of indirect lung injury. Despite a great number of clinical studies, indirect factor trauma/hemorrhagic shock to the function and the mechanism in acute lung injury is not clear yet. Therefore, it is still necessary to carry on relevant analysis in order to thoroughly explore its molecular and cellular mechanisms and the pathway of disease function. In our research, we aimed to identify potential pathogenic genes and do modular analysis by downloading disease-related gene expression profile data. And our dataset is from the NCBI-GEO database. Then, we used the Clusterprofiler R package, GO function, and KEGG pathway enrichment analysis to analyze the core module genes. In addition, we also identified key transcription factors and noncoding RNAs. Based on the high degree of interaction of potential pathogenic genes and their involved functions and pathways, we identified 17 dysfunction modules. Among them, up to 9 modules significantly regulate the response to bacterial-derived molecules, and the response to lipopolysaccharide and other related functional pathways that mediate disease development. In addition, miR-290, miR-30c-5p, miR-195-5p, and miR-1-3p-based ncRNA and Jun, Atf1, and Atf3-based transcription factors have a total of 80 transcription drivers for functional modules. In summary, this study confirmed that miR-30c-5p activates lipopolysaccharide response pathway to promote the pathogenesis of ALI induced by hemorrhagic shock. This result can be an important direction for further research on related deepening diseases such as acute respiratory distress syndrome (ARDS). It further provides a piece of scientific medical evidence for revealing the pathogenic principle and cure difficulty of acute lung injury and also provides important guidance for the design of therapeutic strategies and drug development.

## 1. Introduction

Acute lung injury (ALI) is a clinically complex syndrome involving acute inflammation and microvascular injury and affecting pulmonary vascular and epithelial permeability leading to acute respiratory failure [1]. Among them, trauma/hemorrhagic shock (T/HS) is the main type of indirect lung injury, which drives the release of proinflammatory mediators into the mesenteric lymph (ML) and triggers a systemic inflammatory response and ultimately leads to acute lung injury [2]. The clinicopathological features often present with progressive hypoxemia and respiratory distress, and the deepening of the disease can lead to acute respiratory distress syndrome (ARDS) [1, 3]. At present, there are quite a few medical experts and scholars who have conducted in-depth research on the pathogenesis of T/HS acute lung injury. Recent studies have shown that mesenteric lymph is the main cause of lung injury after T/HS, and its cytokines induce apoptosis of lung endothelial cells and epithelial cells [4]. In addition, the dysregulated inflammation that occurs after severe injury in patients is also caused by intestinal-derived inflammatory mediators carried by the mesenteric lymph. Among them, exosomes belong to extracellular vesicles and serve as an endogenous mediator of immune response, which is released into the mesenteric lymph after T/HS to induce the production of proinflammatory cytokines in macrophages and then participate in the pathogenesis of acute lung injury. It also promotes posttraumatic immune dysfunction by mediating dendritic cell (DC) dysfunction [5]. In an experiment to further explore the pathogenic principle of exosomes, it was important for the activation of macrophages by Toll-like receptor 4 (TLR4). It is worth noting that the cytokines produced by exosome induction can be reversed by TLR4-related pharmacological inhibition [6]. This discovery is highly regarded by scientists such as Sodhi, and the underlying pathogenesis of TLR4 is officially stated. Activation of TLR4 after trauma leads to increased endoplasmic reticulum stress in the intestinal epithelial cells, apoptosis and release of circulating HMGB1, and an increase in the severity of lung injury. Moreover, the wild-type mice lacking TLR4 in intestinal epithelial cells (AEC) did not produce acute lung injury and confirmed its importance for disease development [7]. Interleukin-8 (IL-8) is a potent neutrophil attractant and activator, and its self-forming IL-8 antibody interacts with the Fc*γ*RIIa receptor, which may affect diseases such as neutrophil apoptosis. Mechanism [1]. Moreover, T/HS-induced intestinal and intestinal-induced lung injury also involves complex processes such as intraluminal digestive enzymes, unstirred mucus layer, and systemic ischemia-reperfusion injury [8]. Part of the cause is mediated by a decrease in the level of surfactant protein-D and is associated with apoptosis in alveolar epithelial cells. In terms of biological inhibitors, it was found that the protein level of pulmonary surfactant protein-D returned to normal after administration of activator IL-6, and IL-6 could be used as a prophylactic adjuvant for shock recovery aftershock [9]. Due to the serious harm of the disease, the inhibition mechanism and treatment strategy of T/HS acute lung injury have also been identified by some biologists. Stimulation of the G protein-coupled cell surface receptor A2B adenosine receptor prevents T/HS-induced lung and muscle damage [10]. Tranexamic acid (TXA) is a synthetic derivative of lysine that inhibits T/HS-triggered bronchoalveolar fluid and serum interleukin-6 and TNF-*α* excessive production, and enzymatic activity of myeloperoxidase (MPO) in lung tissue. In addition, TXA treatment partially attenuated the inactivation of the poly ADP-ribose polymerase-1 (PARP1)/nuclear factor *κ*B (NF-*κ*B) signaling pathway in the lungs after T/HS regulation of abnormal lung inflammation [11]. FTY720 can be used as a resuscitation treatment factor to limit T/HS-induced multiple organ dysfunction syndromes (including lung injury, red blood cell damage, and neutrophil perfusion) and T/HS lymphocyte bioactivity [2]. Treatment with CPSI-121 with pharmacological vagal nerve stimulation (VNS) can prevent intestinal barrier failure and attenuate the biological activity of mesenteric lymphocytes, and has potential effects in preventing acute lung injury [12].

RETRACTED

A series of basic experimental studies related to T/HS acute lung injury have carefully analyzed the pathogenesis and treatment models of the disease, but the disease development situation is still grim, and comprehensive and in-depth research is still needed to reveal the underlying disease mechanism that has not yet been elucidated. This study was based on the modular analysis of protein interactions based on microarray expression profiles of T/HS lung injury (experimental group) and T/SS nonlung injury (control group). The resulting miR-30c-5p activates the lipopolysaccharide response pathway to promote the progression of acute lung injury in hemorrhagic shock. It has deepened our understanding of the pathogenesis of T/HS acute lung injury and helps to find biological targets and diagnostic markers for acute lung injury susceptibility after T/HS. At the same time, it is also beneficial to evaluate the risk of acute lung injury and the prognosis of patients with lung injury and also provide a theoretical basis and new strategy for drug development of acute lung injury.

RETRACTED

## 2. Materials and Methods

In the field of immunology, as an important pathogen-related molecular model, it is important to fully understand the toxicity of lipopolysaccharide drugs for effective innate and adaptive immune responses [13]. In this regard, this study also integrated recent reports on the inhibition and treatment of acute lung injury mediated by lipopolysaccharide, both the forsythiaside A (FA) and the acyloxyacyl hydrolase (AOAH) were shown to have an important protective effect on acute lung injury. It improves lung inflammation by interfering with the LPS-TLR4-MyD88-NF-*κ*B signaling pathway and inhibiting the biological activity of alveolar macrophages [14, 15]. The drug liraglutide has been shown to have anti-inflammatory and immunomodulatory effects by inhibiting the NLRP3 inflammasome pathway to alleviate the condition [16]. In addition, many clinical trials have shown that early fluid resuscitation can improve the prognosis of lung injury and reduce the mortality of patients with septic shock. After treatment, it shows effective circulating blood volume and tissue perfusion pressure, improves microcirculation disorder, and increases oxygen partial pressure and oxygenation index [17].

### 2.1. Data Resources

GEO Database (Gene Expression Omnibus) is an internationally recognized public repository of sequential datasets. We collected microarray expression profiles of traumatic hemorrhagic shock (T/HS) model mice, named GSE6332. The data set includes three samples of traumatic/hemorrhagic shock (T/HS) acute lung injury and three samples of traumatic pseudoshock (T/SS) nonlung injury. We then downloaded protein-protein interaction data from the STRING V10 database to construct differentially related PPIs [18].

### 2.2. Differentially Expressed Genes

The differentially expressed genes (DEGs) was analyzed by the limma package [19–21]. The control probe and the probe with low expression were filtered out by quantile normalization. Then, the DEGs in the dataset were identified by default parameters.

### 2.3. High Interaction Module Characterizes the Disequilibrium Mechanisms of T/HS Acute Lung Injury

First, we construct a protein-protein interaction network (PPIs) based on the STING database to observe the high degree of gene interaction and use the ClusterONE [22], a plug-in in the Cytoscape [23] for modularization. These highly interactive modules contain potential pathogenic genes of T/HS acute lung injury, which can best characterize the disorder mechanism and development process of the disease.

### 2.4. Enrichment Analysis

The enrichment analysis was used to explore the potential mechanism of T/HS acute lung injury. In addition, the clusterProfiler [24] was performed to enrich and analyze the GO function and KEGG pathway, respectively, and set *P* value < 0.01 to screen for significant functions and pathways.

RETRACTED

### 2.5. Regulatory TFs and ncRNAs

We scientifically predicted and tested the role of TFs and ncRNAs in T/HS acute lung injury dysfunction module. Regulatory TFs and ncRNAs were defined as significantly affected module genes in the proliferation and metastasis of T/HS acute lung injury cells. *P* value < 0.01 was the screening thresholds.

## 3. Result

### 3.1. Screening for Potential Pathogenic Molecules in T/HS Acute Lung Injury

Biologists conducted many researches on the T/HS ALI and comprehensively summarized a large part of scientific research results in the GEO database. For molecular changes in the course of T/HS acute lung injury, the differentially expressed genes (DEGs) between the experimental and control groups of T/HS ALI were analyzed to obtain a potential disease gene that may cause T/HS acute lung injury. The results showed that we had a total of 1254 differential genes (Table S1). These differential genes have potential effects on the development of T/HS acute lung injury and need further analysis to support it.

### 3.2. Identify T/HS Acute Lung Injury Functional Modules

The interrelationship between differential genes can be observed through a protein interaction network. Then, based on the modular analysis method, these genes clustered expression in PPIs. The clustering of T/HS acute lung injury genes into modules is beneficial to observe the complex interactions among these genes from expression behavior. Finally, we identified 17 T/HS acute lung injury dysfunction modules (Figure 1). The modular analysis of 17 oral tumor height interaction modules, the outer circle of different color dot groups represents the genes of 17 different modules.

### 3.3. High-Level Interaction Module to Characterize Potential Dysfunction of T/HS Acute Lung Injury

GO and KEGG pathway analyses were performed on 17 modules, 28,920 BP terms, 2680 CC terms, and 4520 MF terms and 1354 KEGG pathways were obtained (Table S2, Figures 2(a), 2(b)). These functions were found to focus on biological processes such as the reaction to lipopolysaccharide, the reaction to bacterial-derived molecules, the reaction to metal ions, and the reaction with ruthenium-containing compounds. The enrichment results of the KEGG reflect that the disease-differentiated genes are enriched in amino acid-related pathways such as arginine biosynthesis and phenylalanine metabolism. The high-count results showed that the genes in module 9 significantly regulated the response of the bacterial-derived molecules and the lipopolysaccharide reaction pathway.

RETRACTED

### 3.4. TF and ncRNA Driving T/HS Acute Lung Injury Progression

Transcriptional and posttranscriptional regulation of genes has long been recognized as a key regulator of disease development and progression, while transcription factors and ncRNAs are regulators of common expression and function. Although the regulation of TF and ncRNA on T/HS acute lung injury metastasis has been valued by many biologists. Thus, we performed a pivotal analysis targeted to core functional modules to explore key transcriptional regulators in the regulation of T/HS ALI. A total of four ncRNAs involved four ncRNA-module regulatory pairs (Table S3) and 132 TFs involved 75 TF-module regulatory pairs (Table S4). The above results were introduced into the Cytoscape to display the regulate network (Figures 3(a) and 3(b)). We then analyzed the number of pivoted regulate modules, and ncRNA (miR-290, miR-30c-5p, miR-195-5p and miR-1-3p, etc.) and TF (Jun, Ar and Atf1, etc.) were most regulated. These TFs and ncRNAs may regulate the pathogenesis of T/HS ALI by mediating dysfunctional module genes of T/HS acute lung injury.

## 4. Discussion

Acute lung injury (ALI) caused by traumatic hemorrhagic shock (T/HS) is recognized as a complex clinical acute respiratory syndrome. The measures taken by clinical medicine are still in the early stage of defense, and it is difficult to cope with sudden infections in surgical treatment. Although medical scientists have explored the etiology of T/HS acute lung injury in various aspects, the underlying pathogenesis is still unclear. Based on this, this study explores the process of disease formation through a comprehensive and in-depth analysis of the dysfunction module of T/HS acute lung injury. At the module level, we note that the highly interactive dysfunction module is mainly involved in the reaction of ruthenium-containing compounds, the reaction to corticosteroids, the reaction to organophosphates, the reaction to glucocorticoids, and other inorganic salts and organic compounds. At the same time, up to 9 modules participated in the response to bacterial-derived molecules and the reaction to lipopolysaccharide. Bacterium was important for lung inflammation, and TNF-*α* acts on the recruitment and activation of monocytes in mycobacterial infection. In contrast, mice infected with mycobacteria Bacillus Calmette-Guerin (BCG) without type 1 TNF receptor are prone to cause fatal diseases such as pneumonia [25]. For further investigation of pulmonary infection, [14, 17], Gram-negative bacterial outer membrane lipopolysaccharide (LPS) under the action of the most significant infection, during human inhalation, the dose will be affected dependently causing fever, chills, and bronchoconstriction [26]. It acts as an inflammatory infectious agent mediating pulmonary endothelial barrier dysfunction with reversible cellular deformation and endothelial gap formation [27]. At the molecular level, microRNAs (miRNAs) regulate gene expression during transcription, posttranscription, and inflammatory responses [28]. However, the function in T/HS acute lung injury was unknown. This study is based on hypergeometric testing to identify key miRNAs that regulate core functional modules. Finally, four miRNAs that significantly regulate the progression of T/HS acute lung injury diseases, such as miR-195-5p, miR-30c-5p, miR-1-3p, and miR-290, were obtained. MiR-195-5p is targeted by FGFR1, which mediates apoptosis, in bronchial epithelial cells of chronic obstructive pulmonary disease.

RETRACTED

## 5. Conclusion

Our study explores the process of disease formation through a comprehensive and in-depth analysis of the dysfunction module of T/HS acute lung injury. At the module level, we note that the highly interactive dysfunction module is mainly involved in the reaction of ruthenium-containing compounds, the reaction to corticosteroids, the reaction to organophosphates, the reaction to glucocorticoids, and other inorganic salts and organic compounds.

## Figures and Tables

**Figure 1:** A high-level interaction module to characterize the potential dysfunction of oral tumors.

**Figure 2:** The module gene function and pathway enrichment analysis excerpts. (a) Module gene GO function enrichment analysis excerpt. The color increases from blue to purple, and the enrichment increases significantly. The larger the circle, the greater the proportion of the gene in the module that accounts for the GO function. (b) Module gene KEGG pathway enrichment analysis excerpt. The color increases from blue to purple, and the enrichment increases significantly. The larger the circle, the greater the proportion of the gene in the KEGG pathway entry.

**Figure 3:** The regular network. (a) The regulation of ncRNA pivot regulators on dysfunction modules. The blue circle represents the module. The purple circle represents the ncRNA of the regulatory module. (b) The regulation of the TF pivot regulator on dysfunction modules. The blue circle represents the module. The yellow circle represents the transcription factor of the regulatory module. The size of the circle represents the number of modules that are regulated. The larger the circle, the more the number of controls.

## Data Availability

The datasets used and/or analyzed during the current study are available from the corresponding author on reasonable request.

RETRACTED

## Supplementary Materials

Supplementary 1 Table S1: differential expression of genes in different samples.

Supplementary 2 Table S2: functional and signaling pathway enrichment results of module gene involvement.

Supplementary 3 Table S3: the ncRNA-pivot that regulates modular genes.

Supplementary 4 Table S4: the TF-pivot that regulates modular genes.
